# Analysis of the Efficacy of Acupuncture Combined with Rehabilitation Training in the Treatment of Upper Limb Spasm after Stroke: A Systematic Review and Meta-Analysis

This article has been retracted.

**DOI:** 10.1155/2022/8663356

**Published:** 2022-08-09

**Authors:** Yantan Liao, Fengbin Liu, Jingda Yang, Qishou Ma, Junzhe Li, Yihui Chen, Jiayong Wu

**Affiliations:** ^1^Rehabilitation Hospital Affiliated to Fujian University of Traditional Chinese Medicine, Physical Therapy Department, Fuzhou, Fujian 350003, China; ^2^People's Hospital Affiliated to Fujian University of Traditional Chinese Medicine, Obstetrics and Gynecology Department, Fuzhou, Fujian 350004, China

## Abstract

**Objective:**

Systematic evaluation of the efficacy of acupuncture combined with cognitive rehabilitation training in the treatment of upper limb spasm after cerebral apoplexy.

**Methods:**

The data of CNKI, CBM, CQVIP, Wanfang, and the libraries of Pubmed and Cochrane were searched by computer, and the related literatures about acupuncture combined with cognitive rehabilitation training in the treatment of cognitive dysfunction after stroke were searched. The search time is from January 1, 1995 to January 1, 2022. All data segments were independently analyzed and extracted by two evaluators. After evaluating the quality of the methodology, meta-analysis was carried out by using the RevMan5.4 software.

**Results:**

Finally, 11 studies were included, with a total of 789 subjects. The results of meta-analysis indicated that acupuncture combined with cognitive rehabilitation training was superior to simple cognitive rehabilitation training or drugs in the following aspects, the difference exhibited statistically significant, the total effective rate (RR = 1.58, 95% CI), latency of P300 (MD = −18.46, 95% CI), amplitude of P300 (MD = 1.23, 95% CI (0.82), *P* < 0.00001, 95% CI (0.31)), and activity of daily living (ADL), respectively, were significantly higher compared to the control group (*P* < 0.00001), and the difference was statistically significant (*P* < 0.05). Based on the results of systematic evaluation, the GRADE system recommendation classification method is used to evaluate the quality of evidence. The results show that the level of evidence is low and the intensity of recommendation is weak.

**Conclusion:**

The results of this meta-analysis suggest that the curative effect of acupuncture combined with cognitive rehabilitation training is better compared to simple cognitive rehabilitation training or drugs. However, due to the low quality of the original literature, it needs to be confirmed by multicenter, high-quality, large-sample randomized blind controlled trials in the future.

## 1. Introduction

In the process of stroke recovery, spastic hemiplegia on one side of the limb is one of the common dysfunctions of patients after stroke. Limb spasms not only cause pain but also affect the random movement and standing balance of the patient's limbs. In China, about 65% of stroke patients have muscle spasms on the quadriplegic side. Some patients are even in a state of muscle spasm for a long time, which not only reduces the ability of daily life but also affects the rest and normal sleep of patients [1]. “Apoplexy” appeared as an independent disease name in the Song Dynasty. Chen Wuxue, a physician in the Song Dynasty, put forward “apoplexy” as an independent disease in his “Methodology of extreme Syndromes of three causes-the Theory of Middle Wind” [1, 2]. The main clinical manifestations of stroke are joint flexion but not extension and skin arthralgia but not benevolent, and one side of the limb movement is disadvantageous. For example, for joint flexion and extension, limb movement is not convenient. The word “spasm” is not mentioned in TCM. From the study of clinical symptoms, spasm can be classified as “muscle spasm” in TCM. And there are also specific records about the disease of meridians and tendons in ancient medical books. To trace the origin of the word, “meridian tendons” was first put forward in “Lingshu Jingjin,” and “meridian tendons disease” was put forward as the name of the disease in “difficult Classic.” The first work to record the treatment of meridian tendons disease is “A and B Classic of Acupuncture and moxibustion,” in which there are a large number of words to describe it; the related clinical symptoms mainly include joint movement failure [2]. Until the emergence of the book “Acupuncture and moxibustion Dacheng,” the book not only recorded many methods for the treatment of meridian muscle diseases but also put forward Ashi acupoints and indefinite acupoints and supplemented and summarized the main treatment of its acupoints [3]. In addition, the main occurrence time of tendon arthralgia and corresponding diseases is also put forward in the literature, which is described in the form of words. Jingyue Encyclopedia puts forward the theory of different positions of meridian tendons according to the clinical manifestations, such as follows: “spasm” its disease is in the muscles and veins and then reverse tension [4]. “Spasm” its disease is in the blood and then muscle clonus, in its content, and put forward the specific meaning of “spasm,” and that “spasm” is mainly caused by yin deficiency. Due to the loss of vaginal fluid in the body, moisturizing dysfunction cannot nourish the muscles and veins, and the muscles and veins are anxious, resulting in uncoordinated limb movement or convulsions [4, 5]. In addition, Jingyue Encyclopedia also points out that the occurrence of this disease is also closely related to age, and the elderly are more likely to get sick. The occurrence of spasm is closely related to the twelve meridians. The qi of the twelve meridians gathers in the part of the muscles, which is called the twelve meridians. Human motor function and body development are closely related to meridian tendons. When twelve meridian tendons are invaded by external evil or lost in osmosis, limb relaxation and clonus will occur [5]. In the period of Neijing, the etiological mechanism of stroke is mainly assigned into two aspects, one is internal wind, and the other is external wind.

Acupuncture is a very effective method of TCM in the treatment of limb spasm after stroke [6]. It has been widely adopted in clinic and used in the treatment of stroke sequelae and other chronic diseases. At present, acupuncture therapy, which is mainly used in clinic, not only plays a great role in the treatment of limb spasm after stroke but also has certain advantages in many treatment methods of limb spasm after stroke. Acupuncture can effectively relieve the symptoms of limb spasm after stroke, and it is widely used in clinic, which has its own advantages and significance [6, 7]. With the more in-depth clinical study of limb spasm after stroke, there are more methods for the treatment of limb spasm after stroke, including oral medicine, physiotherapy, and rehabilitation techniques. Comprehensive treatment began to be gradually applied to the clinic, and a single treatment also has its limitations. Combined with the current research situation, it is understood that Western medicine has its unique treatment for limb spasm after stroke, mainly by means of rehabilitation training to enhance limb spasm, while assisting with other ways of treatment, which can effectively prevent muscle atrophy and joint contracture deformation [7]. In traditional Chinese medicine, acupuncture is widely used to treat limb spasm after stroke. Acupuncture treatment of limb spasm after stroke is not only various and convenient to operate, but also recognized by patients because of its remarkable curative effect. Acupuncture has a variety of acupoint selection methods in clinic, including Yangming meridian acupoint selection method, Sanyang meridian acupoint selection method, and the combination of acupuncture and moxibustion with TCM treatment, viscera massage, acupoint injection, physiotherapy, and modern rehabilitation treatment to form a comprehensive therapy. It has also achieved a good therapeutic effect in clinic, and it has been paid more attention by people [8]. In recent years, there are more reports on TCM rehabilitation technology. TCM rehabilitation therapy has been widely adopted in the clinical treatment of limb spasm after stroke [9, 10]. At present, there are few literatures about acupuncture combined with cognitive rehabilitation training in the treatment of upper limb spasm after stroke, but whether it really enhances the therapeutic effect is worth exploring. In order to evaluate its curative effect objectively, this study adopted the Cochrane systematic evaluation method to systematically evaluate and meta-analyze the existing clinical trial results, so as to provide reference for clinical application.

## 2. Patients and Methods

### 2.1. Literature Sources

Chinese National Knowledge Infrastructure (CNKI), China Biomedical Database (CBM), CQVIP Network (CQVIP), Wanfang Database (Wanfang data), Pubmed, and Cochrane Library were searched by computer to find all the comparisons between acupuncture combined with cognitive rehabilitation training and simple cognitive rehabilitation training or drug therapy from January 1, 1995 to January 1, 2021. The retrieval strategy uses the combination of subject words and free words for database retrieval. Chinese retrieval takes CNKI as an example and English retrieval takes Pubmed as an example, as indicated in Table 1.

### 2.2. Literature Inclusion Criteria

The study type of randomized controlled trial (RCT) was limited to Chinese and English, regardless of whether or not blind/distributive concealment was adopted. Repeated published literature was excluded.

#### 2.2.1. Research Object

*(1) Inclusion Criteria*. Inclusion criteria are as follows: (1) to meet the diagnostic criteria adopted by the fourth National Conference on Cerebrovascular Diseases and the criteria for stroke diagnosis and curative effect evaluation formulated by the State Administration of traditional Chinese Medicine [11] and to indicate cerebral infarction or cerebral hemorrhage through cranial CT or craniocerebral MRI, (2) to screen and evaluate patients with cognitive impairment through the cognitive screening record table (CCSE) or with reference to the diagnostic criteria of Petersen [12], (3) there is loss of consciousness or language disorder, and (4) the baseline of the treatment group and the control group is basically the same and comparable.

*(2) Exclusion Criteria*. Exclusion criteria are as follows: (1) severe visual and hearing impairment; (2) severe mental disorder or dementia, epilepsy, and unable to cooperate; (3) accompanied by severe heart, liver, and kidney disease; (4) education level is lower compared to primary school; (5) poor compliance; and (6) cannot tolerate and receive treatment.

#### 2.2.2. Intervention Measures

The treatment group was treated with acupuncture (acupuncture, scalp acupuncture, and electroacupuncture) combined with cognitive rehabilitation training, while the control group was treated with simple cognitive rehabilitation training or drugs.

#### 2.2.3. Outcome Index

(1) The clinical efficacy was the total effective rate, that is, the proportion of the rest except the patients who were ineffective in treatment; (2) the cognitive memory function was assessed by event-related potential P300; (3) the ability of daily living was assessed by ADL scale.

### 2.3. Literature Exclusion Standard

These are the following: (1) cognitive impairment caused by other diseases, (2) only abstracts but lack of full text or incomplete reports of important data and no reply to the author, (3) repeatedly published literature, and (4) the original text is not standard and has obvious errors.

### 2.4. Literature Screening and Data Extraction

The title and abstract of the literature obtained by the two researchers are read independently, and the full text of the literature that may meet the inclusion criteria is read to determine whether it really meets the inclusion criteria. The divergent documents are resolved through discussion or arbitration by a third party, and then, the included documents are extracted according to the contents of the collection table. The collection table includes general information such as author, publication time, number of cases, intervention measures, outcome index, course of treatment, and methodological characteristics such as random method, blind setting, loss of follow-up and withdrawal, and baseline balance.

### 2.5. Document Quality

Evaluation of bias risk assessment included in the study was based on bias risk assessment tools recommended by Cochrane collaboration network [13]. The bias risk assessment included in the study was based on the bias risk assessment tool recommended by Cochrane collaboration network [13]: (1) random allocation method, (2) allocation scheme hiding, (3) participant blind method, (4) analyst blind method, (5) integrity of result data, (6) selectively reported research results, and (7) other sources of bias. Among the above quality standards, if all the standards are “sufficient,” the possibility of various biases is very small, if one of them is “unclear,” there is a moderate possibility of corresponding bias, and if one of them is “inadequate” or “not adopted,” there is a high possibility of corresponding bias. Meanwhile, the quality of the literature was scored by Jadad scale [14], with a total score of 5, 0-2 as low-quality study and 3-5 as high-quality study.

### 2.6. Statistical Analysis Method

The RevMan5 software originated from Cochrane collaboration network for meta-analysis. The mean and standard deviation of the net change difference of serum albumin, prealbumin, and hemoglobin in the experiment, and the control cohorts were input into RevMan5 for analysis. Because the index is a continuous variable, the weighted mean difference (WMD) is used as the effect scale, and 95% confidence interval is selected. First, *χ*^2^ test is used to determine whether there is heterogeneity between the studies; if *P* > 0.05 and *I*^2^ < 50%, it is considered that the included study is homogeneous, and the modified impact model can be collected for meta-analysis. If *P* < 0.05 and *I*^2^ ≥ 50%, when judging the homogeneity of the included study, the combined effect is needed; then, choose the random effect model. If *P* < 0.05, and the source of heterogeneity could not be judged, meta-analysis was not performed, and descriptive analysis was used.

## 3. Results

### 3.1. Search Result

According to the retrieval strategy, a total of 99 related articles were retrieved, 38 repeated articles were excluded, and the remaining 61 articles were left. According to the purpose of the study, inclusion criteria and exclusion criteria, a total of 51 unqualified articles were excluded, and finally, 10 articles were included, all of which were in Chinese. The inclusion process is indicated in Figure 1. In 10 studies, there were 386 cases in the treatment group and 375 cases in the control group, with a total of 761 patients.

### 3.2. The Basic Characteristics of the Inclusion Study (See Table 1 for Details)

#### 3.2.1. Quality Evaluation Included in the Study

In the 10 studies included in this study [10–20], the baseline of patients was analyzed and reported, and the baseline balance was consistent in all studies. There exhibited no significant difference in age, sex, and course of disease between the test group and the control group, and the intervention measures of the test group and the control group were comparable. In terms of random methods, there are 5 studies [11–13, 16, 19] are randomly assigned into groups by using the method of random number table. One study [10] uses the random alphabet method to group randomly; four studies [14, 15, 18, 20] mentioned random grouping, but the specific methods were not explained. One study [17] was randomly assigned into groups according to the order of admission; all studies did not report the blind method and the concealment of allocation schemes; all the literatures did not report loss of follow-up; two studies [11, 13] mentioned the number of withdrawal cases and their reasons; none mentioned whether or not to selectively report the results. The quality of the three studies [11–13] is good, and the possibility of other biases is small. The randomized scheme adopted in one study [17] is problematic and may have other biases. The other six studies are not clear about other biases. The detailed evaluation of methodology quality and the bias risk is indicated in Figures 2(a) and 2(b).

There exhibited no significant difference in age, sex, and course of disease between the test group and the control group, and the intervention measures of the test group and the control group were comparable. In terms of random methods, there are 5 studies [11–13, 16, 19] that are randomly assigned into groups by using the method of random number table. One study [10] uses the random alphabet method to group randomly; four studies [14, 15, 18, 20] mentioned random grouping, but the specific methods were not explained. One study [17] was randomly assigned into groups according to the order of admission; all studies did not report the blind method and the concealment of allocation schemes; all the literatures did not report loss of follow-up; two studies [11, 13] mentioned the number of withdrawal cases and their reasons; none mentioned whether or not to selectively report the results. The quality of the three studies [11–13] is good, and the possibility of other biases is small. The randomized scheme adopted in one study [17] is problematic and may have other biases. The other six studies are not clear about other biases.

### 3.3. Analysis of Outcome Index

#### 3.3.1. Curative Effect Analysis

Of the 10 studies that met the inclusion criteria, 3 [17–19] reported the total effective rate, including 239 cases in the treatment group and 120 cases in the treatment group, total effective 99 cases, control group 119 cases, and total effective 59 cases. The source of the study may be caused by the different control schemes. According to the different control schemes, the patients were assigned into two subgroups, each subgroup had heterogeneity in each outcome index (*P* = 0.03, *I*^2^ = 71%), and the difference was statistically significant (*P* < 0.05). Random effect model was used for meta-analysis. The results indicated that the total effective rate of acupuncture combined with cognitive rehabilitation training was higher compared to the control group, and the difference was statistically significant (RR = 1.58, 95% CI (1.10, 2.26), and *P* = 0.01), and *P* < 0.05 indicates the difference was statistically significant (see Figure 3).

## 4. Discussion

Stroke is a serious threat to the health of human life and has the characteristics of high incidence and high disability rate [19]. Stroke has long been described in traditional Chinese medicine (TCM) in ancient books [20]. But in some cases, limb spasm also has certain benefits to patients, because hemiplegic patients after stroke have to achieve a certain standing balance in the process of rehabilitation, and the spasm of lower limb extensor can help patients maintain their standing posture and walk a short distance. Due to the impairment of limb motor function and disturbance of limb blood circulation, limb edema can occur. Spasm can promote blood reflux to reduce edema of paralyzed limbs and avoid the formation of deep venous thrombosis [21]. Therefore, clinically, we should make good use of the limb spasm which is beneficial to the patient and focus on the treatment of the spasm which is disadvantageous to the recovery of the limb function of the patient. Limb spasm after stroke not only reduces the quality of life of patients but also hinders the follow-up rehabilitation of patients with limb spasm after stroke, which is the key factor affecting the follow-up rehabilitation of patients with limb spasm after stroke. Therefore, what kind of treatment to enhance the state of limb spasm and how to promote the clinical efficacy of the treatment of limb spasm after stroke is a problem that needs to be studied in contemporary medical circles [22].

Clinically, spasm refers to intermittent or continuous involuntary contraction of muscles or muscle groups, mainly due to the injury of upper motor nerve cells and transmission disorders of the nervous system, resulting in clinical symptoms of spastic hemiplegia. The cerebral cortex is the superior center of the human nervous system. The signal is transmitted between the brain and the spinal cord, centered at the bottom of the spinal cord, and the reflexes of motoneurons are regulated by superior motoneurons [23]. When normal people are clear-headed, their body and various parts of the muscles will maintain a certain sense of tension, and this state is called muscle tension, referred to as muscle tension. The generation and maintenance of muscle tone is accomplished by a reflex arc called “*γ*-loop.” The reflex arc of the “*γ*-loop” passes into the stimulus signal through two kinds of receptors. Even if you rest calmly, the muscles will not relax and the muscle tension will not disappear [24]. In terms of muscle tone, it is mainly regulated by the central system, and it can inhibit muscle tension to a certain extent in the corresponding structures above or above the midbrain, while in the reticular structure of the ventral part of the medulla oblongata below the midbrain, it is the main muscle tension inhibition area, and the main function of this part is to reduce muscle tension, and the vestibular system itself also plays a role, which can facilitate muscle tension. Therefore, it will directly or indirectly affect muscle tone [25]. In addition, there are a variety of neurotransmitters in the central nervous system, and the neurotransmitters that play an important role in the formation of spasm are amino acid neurotransmitters. Amino acid neurotransmitters can also be assigned into different categories: one is excitatory amino acid, mainly the following: glutamic acid, aspartate. The other is mainly inhibitory amino acids, which are widely distributed in the central system of the human body and are also the most important inhibitory neurotransmitters in the brain or bone marrow, which cannot be ignored in the human body [25, 26]. In addition, to a certain extent, the suppression of muscle stretch reflex function will first lead to delayed paralysis, with the passage of time, the recovery of stretch reflex, the main recovery of the lower limb extensor reflex, the muscle spindle is still in a higher sensitive state to the stretch reflex, so the fibers in the muscle spindle are activated for a long time (anterior stretch), and the stretch response to muscle tissue is especially rapid and sensitive. Neu et al. made a specific analysis in the course of the study and concluded that there is a proportional relationship between muscle tone rating and Mmax and Mslp, and it shows a positive proportional relationship, so the proportional relationship between Mmax and Msl can be adopted as the main sign to evaluate the specific state of spasm [26]. Modern medical research also found that the essence of meridian tendon is similar to the theory of myofascial chain, and there are many similarities in its diagnosis and treatment. The essence of meridian tendons is the muscular system and nervous system [27].

In TCM, it is believed that the wind mainly enters the human body from outside the human body, and the spasm after stroke is mainly caused by external factors, that is, the wind. The Yellow Emperor's Internal Classic [28] records: “the wind is the strength of all diseases, and the number of good deeds changes.” Wind evil is the main factor at the beginning of all diseases. Wind evil is easy to attack the human body and is caused by other evil qi. The influencing factors of wind are not fixed. If people are affected by wind evil and lead to stroke, they can be assigned into different meridians. The pathogenic characteristics of wind evil are also listed in the literature. Meanwhile, it is also specifically described that wind evil can be combined with cold evil and heat evil to produce disease. “Ming doctor refers to” records, people after a stroke due to wind attack, and there will be corresponding symptoms, such as limb paralysis or mouth and eye askew. In serious cases, it will be inconvenient to move, and it may also lose the ability to move. The main cause is that wind pathogenic dampness and toxin remain in the meridians of the whole body, resulting in obstruction of meridians and qi stagnation at the ends of the limbs, so the limbs are restless and treated with Huoluo Dan. Deficiency of vital qi, invasion of evil qi into human body and blocking of meridians and collaterals are the main internal factors reflected by limb spasm after stroke, which are also recorded in the literature [29]. It is pointed out in the literature that “this is caused by deficiency of the body, and the evil of the wind lies in the muscles.” If the limbs cannot flex and extend normally, it is likely to be caused by the deficiency of the body, and the evil of the wind invades between the muscles and bones. While the evil of wind is a very important factor leading to spasm of one side of the limb, it can be concluded that people with weaker physique are vulnerable to limb spasm because of their own deficiency of upright qi [29, 30]. The Medical Classics will solve. Stroke also has the following records: “if the five internal organs are sick and maladjusted at 04:00, then evil qi will enter the disease by taking advantage of the deficiency.” The damage to the five internal organs, the imbalance of qi at 04:00, the deficiency of vital qi in the human body, and the failure of reason are not closed. Therefore, the spasm phenomenon after stroke is due to the wind evil invading the muscles and veins of the limbs, resulting in the discomfort of meridian qi, and the appearance of the main symptom of meridian spasm. There are also specific records in ancient Chinese literature, pointing out that the Zang-fu organs related to tendon clonus are the liver. Meanwhile, it is also clearly pointed out in ancient Chinese medicine that the liver plays an important role in tendon, and wind evil will harm the muscles and veins of the human body under certain conditions [30]. In TCM, it is believed that the occurrence of spasm is mainly due to the injury of evil qi to the liver and the main tendon of the liver, and there is a close relationship between them, and there are many descriptions of wind evil in the literature. Some physicians think that yin deficiency of liver and kidney is the fundamental pathogenesis of limb spasm after stroke [31]. Some scholars also put forward the following point of view, which believes that the main pathogenesis of stroke spastic hemiplegia is caused by the weakness of yang qi, the main accumulated viscera of yang deficiency is spleen and stomach, spleen deficiency produces dampness, and dampness hinders blood flow, resulting in blood stasis, blood stasis block meridians, meridians are blocked, and spasms occur [32].

For the rehabilitation treatment of limb spasm after stroke, the commonly adopted clinical methods are drug therapy, physiotherapy, occupational therapy, and characteristic treatment of TCM [32, 33]. The characteristic diagnosis and treatment methods of TCM, such as acupuncture, collapse, TCM, massage, bubble washing, and acupoint application, are widely adopted in the treatment of spasm after stroke, while the treatment of TCM has the characteristics of strong pertinence, stable, and exact curative effect. Therefore, traditional Chinese medicine has great advantages in the treatment of limb spasm after stroke, which can reduce the degree of spasm and promote the recovery of limb dyskinesia. However, there are also some problems, such as the superposition of a variety of effective treatment methods, lack of theoretical guidance, and lack of clinical evidence. Compared with the systematic TCM rehabilitation project, the maneuverability is getting worse and worse. Therefore, it is necessary to establish a standardized and effective TCM rehabilitation program under the guidance of systematic TCM theory [33]. The main acupuncture methods used in clinic are as follows: (1) according to the acupuncture site, it can be assigned into abdominal acupuncture, eye acupuncture, and body acupuncture; abdominal acupuncture is mainly through acupuncture at some acupoints in the abdomen of the human body; it can not only achieve the main effect of soothing the liver and regulating qi but also regulate the body and mind and play an important role in the recovery of Zang-fu function [34]. In addition, acupuncture at some acupoints in the abdomen can also ensure the patency of human blood, which is conducive to the recovery of limb function as soon as possible. Takeda and Kawamura in the course of the study put forward the following conclusions; they believe that there are two main methods for the treatment of spastic hemiplegia after stroke, abdominal acupuncture, and body acupuncture, respectively, which have corresponding effects on the treatment of spastic hemiplegia [35]. The clinical therapeutic effect of abdominal acupuncture is better compared to body acupuncture. Eye acupuncture is mainly through the use of acupuncture to stimulate some acupoints around the eyes; in this process, it can achieve the effect of disease treatment. According to Cheng et al., the combination of eye acupuncture and wax therapy is used to treat limb spasm after ischemic stroke [36]. The results demonstrate that the treatment of eye acupuncture combined with wax therapy is better compared to simple wax therapy in improving patients' ability of daily life and motor function; (2) the methods of acupuncture can be assigned into two kinds, the first is yin-yang reinforcing and reducing needling, and the second is three tonifying and reducing needling. Shoutai investigated and analyzed the method of tonifying and reducing yin and yang as the treatment group and the conventional acupuncture method as the control group [37]. After a period of clinical study, the actual situation of limb spasm of stroke patients was observed, and the muscle tension, motor function, and activities of daily living before and after treatment were compared and analyzed. After intervention, the degree of limb spasm in both groups was improved, suggesting that the two acupuncture methods play an important role in improving the ability of daily life of patients. However, the curative effect of yin-yang tonifying and purging method is more effective than conventional acupuncture method. Varjassy made a scientific analysis in the process of investigation, which mainly compared the three tonifying and three purging acupuncture methods with conventional acupuncture methods, and also focused on recording its specific therapeutic results on limb spasm after stroke [38]. The results demonstrate that compared with the traditional acupuncture method, the three-tonifying and three-purging acupuncture method has a better clinical therapeutic effect on limb spasm after stroke. Combined with the current research, doctors also gave a unified overview of the etiology and mechanism of limb spasm after stroke, which is mainly caused by the dysfunction of liver and spleen.

Liu et al. believe that simple rehabilitation training has a certain effect on the recovery of spasticity of upper limbs after stroke, but it is relatively slow [39]. Meanwhile, they also mentioned that acupuncture can dredge the meridians and collaterals of spasms of upper limbs, make the blood circulation of the affected limbs smooth, and thus enhance the spasmodic state of the affected limbs. Through the study, it is proved that acupuncture combined with rehabilitation exercise is more effective than simple acupuncture and simple rehabilitation exercise. According to modern medicine, direct brain injury or reduction of regional cerebral blood flow caused by stroke leads to insufficient cerebral blood supply, leading to chronic cerebral ischemia and hypoxia, neurofunctional degeneration, nerve cell degeneration, softening, and atrophy, affecting structural basic cognition [39, 40]. Acupuncture can obviously protect against cerebral ischemic injury, improve cerebral blood flow, promote the establishment of collateral circulation in cerebral necrotic area, activate nerve cell and nerve fiber regeneration, enhance brain cell ischemia and hypoxia, and finally affect the smooth flow of memory loop [40]. Through rich stimuli such as sight, touch, and hearing, cognitive rehabilitation training can enhance patients' orientation ability, visual spatial resolution, master specific skills and techniques, give full play to compensatory memory, and strengthen the ability to analyze and deal with problems. Meanwhile, acupuncture and cognitive rehabilitation training, as a special peripheral sensory input, can adjust the excitability of each motor neuron in the neural reflex loop and realize the functional reorganization and compensation of the cerebral cortex. So that the cognitive impairment of stroke patients can be enhanced. Therefore, the organic combination of the two therapies can reduce the damage of cerebrovascular disease to cognitive function to a great extent, promote cognitive function, and thus strengthen the quality of life of patients. A total of 11 randomized controlled trials were included in this systematic review, with a total of 789 patients. The results of meta-analysis also indicated that acupuncture combined with cognitive rehabilitation training in the treatment of cognitive impairment after stroke was superior to simple cognitive rehabilitation training or drug therapy in clinical efficacy, P300 measurement and activities of daily life, and the difference exhibited statistically significant. However, in view of the low quality of the original research included in this meta-analysis, which affects the authenticity of the conclusions and based on the GRADE system, the quality of evidence and the recommended level is 2C, so clinicians are advised to choose carefully. In addition, this study has some limitations, all of which do not explain the use of blind method, no mention of distributive concealment and intention to treat (ITT) analysis, and the quality is low; all studies are domestic literature, lack of foreign literature, and there is a large language bias, which may affect the conclusion and extrapolation of meta-analysis. In the original study, small sample size, different course of disease, different intervention time, evaluation criteria, and evaluation time were slightly different, which had a certain impact on the evaluation results, thus affecting the results and argumentation intensity. The same idea can be found in the study put forward by Xu et al.[41]. They have applied new methods in the study, and the conclusions drawn can also give some support to this study. There are some limitations in this study. First of all, the sample size of the references included in this study is small, and they all belong to single-center research; there is a certain deviation. In the future research, we will carry out a large sample of prospective studies and hopefully draw more valuable conclusions.

The results of this meta-analysis suggest that the curative effect of acupuncture combined with cognitive rehabilitation training is better compared to simple cognitive rehabilitation training or drugs. However, due to the low quality of the original literature, it needs to be confirmed by multicenter, high-quality, large-sample randomized blind controlled trials in the future.

## Figures and Tables

**Figure 1:** Document retrieval process.A total of 99 related articles were retrieved, 38 repeated articles were excluded, and the remaining 61 articles were left. According to the purpose of the study, inclusion criteria and exclusion criteria, a total of 51 unqualified articles were excluded, and finally, 10 articles were included, all of which were in Chinese. The inclusion process is indicated in Figure 1. In 10 studies, there were 386 cases in the treatment group and 375 cases in the control group, with a total of 761 patients.

**Figure 2:** (a, b) The detailed evaluation of methodology quality and the bias risk in this study.

**Figure 3:** Curative effect analysis in this study.Of the 10 studies that met the inclusion criteria, 3 [17–19] reported the total effective rate, including 239 cases in the treatment group and 120 cases in the treatment group, total effective 99 cases, control group 119 cases, and total effective 59 cases. The source of the study may be caused by the different control schemes. According to the different control schemes, the patients were assigned into two subgroups, and each subgroup had heterogeneity in each outcome index (*P* = 0.03, *I*^2^ = 71%), and the difference was statistically significant (*P* < 0.05). Random effect model was used for meta-analysis. The results indicated that the total effective rate of acupuncture combined with cognitive rehabilitation training was higher compared to the control group, and the difference was statistically significant (RR = 1.58, 95% CI (1.10, 2.26), *P* = 0.01), and *P* < 0.05 indicates the difference was statistically significant.

**Table 1:** The basic characteristics of the inclusion literatures in this study.

Included in the study	Intervention measures	Sample size	Outcome index
Ma Jiaying	Simple rehabilitation training Acupuncture combined with rehabilitation training	74	SF-MA scoring
Li Chuang	Rehabilitation treatment Rehabilitation combined with acupuncture	74	(SF-MA) scoring and Bathel Index (BI)
Song Wuhui	Routine drug therapy and nursing; acupuncture treatment and comprehensive rehabilitation training	118	Ashworth spasm score
LV Wanjuan	Acupuncture combined rehabilitation training Treatment of rehabilitation training	80	Curative effect
Yang Xuemei	Warming acupuncture and moxibustion Acupuncture treatment	60	Ashworth scale scoring, simplification Fugl-Meyer Motor function score (upper limb), Barthel Index
Zhang Kui	Western medicine treatment+rehabilitation training Acupuncture therapy of TCM combined with rehabilitation training	40	Ashworth, evaluation of motor function of upper limb (FMA), assessment of self-care ability in daily life (FCA scoring)
NiHuanHuan	Acupuncture at Jing acupoint and self-made Shangjie spasm acupoint+rehabilitation training Simple rehabilitation training therapy	100	Improvement Ashworth, evaluation of motor function of upper limb (FMA), assessment of self-care ability in daily life (FCA scoring)
Zhang Ling	Routine rehabilitation training On this basis, it is treated with acupuncture and moxibustion of TCM	80	SF-MA scoring
Cai Yisheng	Rehabilitation treatment On the basis of the control group, combined with acupuncture and moxibustion treatment	74	SF-MA scoring and Bathel Index (BI) score
Chang Jingjing	Warm acupuncture and moxibustion treatment Routine acupuncture treatment	60	Improvement Ashworth Rating scale, simplify Fugl-Meyer Motor function score scale
